# A Novel COVID-19 Diagnosis Support System Using the Stacking Approach and Transfer Learning Technique on Chest X-Ray Images

**DOI:** 10.1155/2021/9437538

**Published:** 2021-11-05

**Authors:** Soufiane Hamida, Oussama El Gannour, Bouchaib Cherradi, Abdelhadi Raihani, Hicham Moujahid, Hassan Ouajji

**Affiliations:** ^1^SSDIA Laboratory, ENSET of Mohammedia, Hassan II University of Casablanca, BP 159, Mohammedia, Morocco; ^2^STIE Team, CRMEF Casablanca-Settat, Provincial Section of El Jadida, 24000 El Jadida, Morocco

## Abstract

COVID-19 is an infectious disease-causing flu-like respiratory problem with various symptoms such as cough or fever, which in severe cases can cause pneumonia. The aim of this paper is to develop a rapid and accurate medical diagnosis support system to detect COVID-19 in chest X-ray images using a stacking approach combining transfer learning techniques and KNN algorithm for selection of the best model. In deep learning, we have multiple approaches for building a classification system for analyzing radiographic images. In this work, we used the transfer learning technique. This approach makes it possible to store and use the knowledge acquired from a pretrained convolutional neural network to solve a new problem. To ensure the robustness of the proposed system for diagnosing patients with COVID-19 using X-ray images, we used a machine learning method called the stacking approach to combine the performances of the many transfer learning-based models. The generated model was trained on a dataset containing four classes, namely, COVID-19, tuberculosis, viral pneumonia, and normal cases. The dataset used was collected from a six-source dataset of X-ray images. To evaluate the performance of the proposed system, we used different common evaluation measures. Our proposed system achieves an extremely good accuracy of 99.23% exceeding many previous related studies.

## 1. Introduction

The SARS-CoV-2 has caused the borders of many countries to be closed and millions of citizens to be confined to their homes due to infection rates; there have been more than 147 million confirmed cases worldwide at this time (April 25, 2021). This virus originated in China in December 2019. At that time, China succeeded in containing the virus for almost three months after the start of the crisis. As of March 2020, Europe was the focus for the germination of the virus, where it infected more than 445000 people [1,2]. Italy became the country which recorded the highest death toll, followed by Spain, which overtook the Asian countries in death toll. This number is continuously increasing. Clinical features of infected COVID-19 cases include fever, respiratory symptoms, cough, dyspnea, and viral pneumonia [3]. The COVID-19 test is based on taking samples from the respiratory tract [4]. A high number of tests may prove to be the key tool to stop the virus spread in some countries. However, it is important to find and develop alternative methods to perform these tests quickly and efficiently.

Artificial Intelligence (AI) techniques have been widely used in many applications such as handwriting recognition [5], rumors or fake news detection in social media [6,7], medical diagnosis support systems (MDSS) [8,9], prediction of patients with heart disease [10–14], and MRI image segmentation [15–21]. Particularly in the medical field, these techniques have been proved invaluable in predicting positive cases of multiple diseases [14,22]. In the context of the COVID-19 pandemic spread, AI techniques have gained particular interest in terms of predicting positive cases based on different medical data. In addition, many computer-aided diagnosis (CAD) systems based on AI techniques for COVID-19 prediction using principally chest X-ray as input data have been proposed [23–27].

The main contribution of our paper is to propose and implement a novel architecture of an automatic detection system as an alternative diagnostic option to prevent the coronavirus spread [28]. This study is based on the combination of six different sources of X-ray image datasets. From these datasets, we generate a new radiographic image dataset containing four classes, namely, normal, COVID-19, tuberculosis, and pneumonia. The application of image processing allows image standardization and improves model learning.

Furthermore, we aim to improve the prediction accuracy of COVID-19. Thus, the proposed system combines five transfer learning (TL) algorithms, namely, ResNet152V2, ResNet101V2, MobileNetV2, VGG16, and VGG19. These TL-based models automatically extract the radiographic images' features. Then, we implemented the stacking technique and the KNN algorithm to combine the performances of the five generated classifiers models and make the final prediction. Indeed, this method can help choose the best model to detect patients infected with COVID-19. The main contribution of this paper consists of the development of an accurate medical diagnosis support system to detect COVID-19 in chest X-ray images using a stacking approach combining transfer learning techniques and KNN algorithm for the choice of the best model. To reach this objective, we trained and tested the proposed system on a consistent dataset of normal, viral pneumonia, tuberculosis, and COVID-19 cases. Then, the best generated model was compared with some models from the literature. Finally, the obtained results in terms of common metrics were compared to the state-of-the-art models.

The rest of this paper is organized as follows: Section 2 presents some relevant related work.  Section 3 describes the materials and methods used, the dataset used, and TL algorithms and methodology followed. Experimental results and discussion are given in Section 4. Finally, we conclude our work in Section 5 with some future perspectives.

## 2. Review of Some Related Works

In the last year, researchers have developed and published many works with the goal of combating the SARS-CoV-2 global pandemic [29–32]. In the field of diagnosis, many studies used Artificial Intelligence techniques to process X-ray images and detect the effect in terms of percentage of the virus in a patient's lungs. Deep learning approaches are the most frequently used in image classification to achieve better results than those using traditional ML approaches [33]. In this section, we limit our investigation to some research using TL technique-based models to diagnose COVID-19 [34].

In [35], the ResNet50 network-based deep transfer learning model achieved 93.01% accuracy for a binary classification of cases with and without COVID-19. This model uses CT type images taken from two open-source datasets.

Other research proposes a new architecture for the detection of cases infected by COVID-19 called CovXNet [36]. This architecture is based on a deep CNN. The authors used 5,856 chest X-ray images composed of four classes: COVID-19, normal, viral pneumonia, and bacterial pneumonia. The CovXNet model achieved an accuracy of 89.6% for 3 classes and 90.6% for 4 classes.

Another model called CoroNet presented in [37] proposes a deep convolutional network, based on the Xception architecture. This model was trained on radiographic images collected from two public databases. This model reached a classification accuracy of 99% for 2 classes, 95% for 3 classes, and 89.6% for 4 classes.

A comparative study published in [38] presented a system based on 10 transfer learning-based models, namely, AlexNet, VGG16, VGG19, SqueezeNet, GoogLeNet, MobileNetV2, ResNet18, ResNet50, ResNet101, and finally Xception. The models trained on a database containing two classes: COVID-19 and viral pneumonia. The authors concluded that ResNet101 is the best model for the reliable detection of COVID-19 with an accuracy of 99.51%.

The proposed study in [39] uses various deep learning architectures such as VGG16, DenseNet121, Xception, NASNet, and EfficientNet, to develop a diagnosis support system of COVID-19. The dataset used contains three classes, and the highest accuracy obtained was 93.48% by EfficientNet.

In [40], the authors proposed a model based on AlexNet architecture for feature extraction and classification of the X-ray images. They used a strength Pareto evolutionary algorithm-II (SPEA-II) to select the best hyperparameters for this model. The proposed model reached an accuracy of 99.13% with a multiclass database.

Another study published in [41] proposed a diagnostic system based on the majority voting method according to the results given by five classifiers: MobileNetV2, ResNet50V2, ResNet50V1, DenseNet201, and ResNet11. This system is based on X-ray image dataset with the three classes of COVID-19, viral pneumonia, and normal. The best accuracy obtained by this model was 99.31%.

In [42], the authors proposed an automated diagnostic model of chest X-rays involving COVID-19. The proposed model uses the truncated DenseNet network based on TL, partial layer freezing, and feature fusion named Fused-DenseNet-Tiny. The proposed model reached a maximal accuracy of 97.99% with only 1.2 million parameters.

In [43], the authors proposed a deep learning model based on pretrained models using majority voting. To build this model, open-source chest X-ray images of normal, pneumonia, and COVID-19 cases were used in this study. The proposed model achieved an accuracy of 99.26%.

Other research published in [44] offered three pretrained models for building a diagnostic system: ResNet50V2, VGG16, and Inception V3. For this study, the dataset used was obtained from two publicly available data sources, containing three classes: COVID-19, normal, and pneumonia X-ray images. The best accuracy achieved by this model was 95.49%.

In [45], The VGG16 network based on transfer learning model achieved an accuracy of 91.69% in a multiclassification of COVID-19-infected, normal, and pneumonia cases. The model proposed in this study is based on X-ray images from a publicly available dataset.

In [46], three pretrained transfer learning models were proposed: VGG16, Inception V3, and lastly EfficientNetB0. COVID-19, normal, and viral pneumonia X-ray images were the three classes in the dataset used in this study, which was compiled from a variety of public sources. For VGG16, Inception V3, and EfficientNetB0, the accuracy of the proposed models was 87.84%, 91.32%, and 92.93%, respectively.  Table 1 summarizes these works by citing the number of classes, the models used, and the best reached values in terms of evaluation metrics.

## 3. Materials and Methods

### 3.1. Global Overview on the Proposed COVID-19 Diagnosis System

In this paper, we proposed a diagnosis system based on stacking technique using various TL models for detecting patients infected with COVID-19. We selected five powerful TL models available in the Keras library. The dataset used was based on six-source databases containing chest X-ray images. From these datasets, we generated a new database with four classes, normal, COVID-19, pneumonia, and tuberculosis [47]. Furthermore, we split the dataset obtained into three parts, training set, validation set, and testing set. Then, we started by applying a series of preprocessing steps to the dataset images. All the chest X-ray images were normalized to the same dimension of 224 × 224 × 3.

The training step involves two levels to generate the final model. The first training level is the Base-Models as the well-known models in TL, namely, ResNet152V2, ResNet101V2, MobileNetV2, VGG16, and VGG19. These models take as input the training set with a default dimension of 224 × 224 × 3. Moreover, we define and detail in Section 3.4 the parameters of each proposed TL-based model. After building the models, we used a validation set to avoid overfitting or underfitting problems. Then, we used the testing set to classify and predict classes. The output prediction obtained in the first training level would be used as input at the metalevel. In the second level of the training phase, we applied the stacking technique to combine the predictions made by each classifier. This technique used the KNN algorithm [48–50], to make the final prediction by contributing to the performance of Base-Models. Finally, we saved the generated model and evaluated the proposed model performance.  Figure 1 describes the main stages of building a COVID-19 diagnosis system architecture.

### 3.2. Stacking Technique

Stacking is one of the most frequently used ensemble methods in ML. The overall idea of this technique is to build many models with completely different algorithmic program types to achieve a final prediction. This method uses another algorithm to learn how to combine predictions from various ML algorithms [51]. Therefore, the input for this final algorithm is the prediction outputs of these various base algorithms. The input of this model is an ensemble which includes *n* classification models.  Figure 2 shows the steps followed to apply the stacking technique.

### 3.3. Dataset Description

As mentioned before, this work relied on the exploration of six different sources of chest X-ray image datasets. In Figure 3, we present some samples from these datasets.

A diversity of datasets allowed us to increase the size of the dataset used in this study. In addition, this will ensure an improvement in terms of detection performance.  Table 2 summarizes all the datasets explored in order to generate a final dataset containing four classes: COVID-19, tuberculosis, viral pneumonia, and normal.

After preparing our dataset, we split it into three parts as follows: 80% for training, 10% for validation, and 10% for testing. The images used in this study did not have fixed dimensions as all came from various reliable sources. For this, we proceeded to resize and normalize all X-ray images to 1024 × 1024.  Table 3 represents the distributions of the dataset images by class.

### 3.4. Tuned Pretrained Models Based on TL Technique

#### 3.4.1. Tuned ResNet152V2-Based Model

The original version of ResNetV2 convolutional neural network (CNN) architecture contains two models, namely, ResNet152V2 and ResNet101V2. These models were developed by Microsoft Research Asia (https://www.microsoft.com/en-us/research/lab/microsoft-research-asia/) based on the ResNetV1 (https://github.com/tensorflow/models/blob/master/research/slim/nets/resnet_v1.py) model in 2016, with different optimizers for each layer to improve the accuracy. In this work, we used ResNet152V2 that reached an accuracy of 94.2% based on the ImageNet dataset. Accordingly, we added some convolutional, flatten, and dense layers after the original version. The architecture details of the proposed tuned version based on ResNet152V2 are presented in Table 4.

The architecture consisted of 70525188 total parameters, with 70381444 trainable parameters and 143744 nontrainable parameters.

#### 3.4.2. Tuned ResNet101V2-Based Model

The second model from the ResNetV2 family is ResNet101V2. This CNN model was formed on the ImageNet dataset. In addition, it reached an accuracy of 93.8%.  Table 5 illustrates the architecture details of this tuned model.

The architecture consisted of 54820100 total parameters, with 54722436 trainable parameters and 97664 nontrainable parameters.

#### 3.4.3. Tuned MobileNetV2-Based Model

The MobileNetV2 model is a CNN containing 53 layers with a depth of 88. Developed in 2018 and trained on a million images from the ImageNet database [52], it reached an accuracy of 90.1% for this dataset.  Table 6 represents the model complexity of our proposed tuned architecture.

The architecture consisted of 13665092 total parameters, with 13930680 trainable parameters and 34112 nontrainable parameters.

#### 3.4.4. Tuned VGG16-Based Model

VGG16 is a CNN model proposed by a team of researchers from the University of Oxford. Trained on ImageNet database, the model achieves 90.1% accuracy.  Table 7 illustrates the complexity details of the proposed tuned model.

The architecture consisted of 17469508 total parameters, with 17460508 trainable parameters and 0 nontrainable parameters.

#### 3.4.5. Tuned VGG19-Based Model

VGG19 is a CNN model that was created in 2015. This model is trained on a million images from the ImageNet database with a depth of 26. It reached an accuracy of 90% with this dataset. In Table 8, we present the proposed tuned architecture based on VGG19 model.

The architecture consisted of 22779204 total parameters, with 22779204 trainable parameters and 0 nontrainable parameters.

## 4. Results and Discussion

Before presenting our results and findings, we first present in the following section some common performance evaluation techniques that are usually used to evaluate ML models at training and testing stages. We start by drawing the confusion matrix and calculating some evaluation metrics. This section presents the metrics and the experimental results obtained by studied models. The confusion matrix allows evaluation of the obtained classification.

### 4.1. Confusion Matrix and Performance Evaluation Measures

In classification problems, a confusion matrix is a table with two dimensions: reference and predicted. This table is used to classify the prediction obtained by classifiers. Moreover, the confusion matrix has identical sets of classes in each row of its dimension. This can allow verifying the confusion between the different classes by calculating four elements, namely, True Positive (TP), False Positive (FP), True Negative (TN), and False Negative (FN) [53]. The confusion elements for each class *ClassX* are given by the following equations:

(1) $$\begin{array}{c} {\text{TP}}_{\text{ClassX}}=C_{i,i},\\ {\text{FN}}_{\text{ClassX}}=\overset{4}{\underset{l=1}{\sum }}C_{i,l}-{\text{TP}}_{\text{ClassX}},\\ {\text{FP}}_{\text{ClassX}}=\overset{4}{\underset{l=1}{\sum }}C_{l,i}-{\text{TP}}_{\text{ClassX}},\\ {\text{TN}}_{\text{ClassX}}=\overset{4}{\underset{l=1}{\sum }}\overset{4}{\underset{k=1}{\sum }}C_{l,k}-\left({\text{FP}}_{\text{ClassX}}+{\text{FN}}_{\text{ClassX}}+{\text{TP}}_{\text{ClassX}}\right), \end{array}$$

where *C*_i,i_ is the number of samples correctly classified for a given class, *C*_i,l_ is the number of negative samples that are confused with another class, *C*_l,i_ is the number of positive samples that are confused with another class, and *C*_l,k_ is the sum of all samples.

We calculated five scoring metrics used in this study: the accuracy, precision, sensitivity, specificity, and negative predictive value (NPV). These metrics are given by the following equations:

(2) $$\begin{array}{c} \text{accuracy}=\frac{\mathrm{TP}+\mathrm{TN}}{\mathrm{TP}+\mathrm{TN}+\mathrm{FP}+\mathrm{FN}},\\ \text{precision}=\frac{\mathrm{TP}}{\mathrm{TP}+\mathrm{FP}},\\ \text{sensitivity}=\frac{\mathrm{TP}}{\mathrm{TP}+\mathrm{FN}},\\ \text{specificity}=\frac{\mathrm{TN}}{\mathrm{TN}+\mathrm{FP}},\\ \text{NPV}=\frac{\mathrm{TN}}{\mathrm{TN}+\mathrm{FN}}. \end{array}$$

### 4.2. Experimental Results

In this section, we present the main experimental results obtained from this study. Firstly, we show the training results by plotting the accuracy and loss curves for all models used. Then, we draw the confusion matrix for each model.

#### 4.2.1. Training of CNN Model Results

In this study, we used the TensorFlow 2.1 library (https://www.tensorflow.org/) to import the original pretrained models and implement the proposed tuned models based on TL technique. We used the library's default Python API. Models were instantiated using the default implementation of Keras (https://github.com/fchollet/keras). Regarding the combination of model performances, we implemented the stacking method in Python language. We used the Scikit-Learn Library (https://scikit-learn.org/stable/) for KNN models. All the experiments were executed in Python language, and we used Jupyter library for easy evaluation of the results. Furthermore, we used the online Google Colab platform to train the proposed TL-based models. Note that Google Colab is a cloud service based on Jupyter Notebook for training and researching the algorithms of ML and DL. This platform used Tesla K80 GPU with 12 GB of GDDR5 VRAM, Intel Xeon Processor with 2 cores @ 2.20 GHz and 13 GB RAM. For all the algorithms used, we performed the training using the Adam optimizer and the cross-entropy loss function. The input image sizes for all arrays are 224-by-224 pixels.  Table 9 presents the hyperparameters used to tune the Base-Models used in this study.

We trained all Base-Models, ResNet152V2, ResNet101V2, MobileNetV2, VGG16, and VGG19, across 25 epochs with the same configuration to ensure comparable results. In Figure 4, we present the plots of accuracy and loss function of the five studied classifiers. The plots are drawn for the training and the validation sets of our chest X-ray datasets containing four classes.

Generally, these curves represent epochs on the *x*-axis and improvement on the *y*-axis. The training curve gives an idea about the successful model training. It is computed from the training set. In fact, 25 epochs were sufficient for all the models to converge. The validation curve provides an idea as to whether the model is underfitting, overfitting, or just right for some ranges of hyperparameter values. However, more epochs were needed to reach the convergence stage, especially for VGG19 and VGG16. Moreover, the overfitting degree was weak in all models. Indeed, the convergence of the accuracy on the training set is close to its convergence on the validation set. From these curves, we concluded that all the models reached an accuracy of 98% during the validation phase. However, the VGG19 model achieves an accuracy value equal to 99.13%. From the loss curves, we noticed that the average loss value for all these models equals 0.1%.

#### 4.2.2. Testing of the Proposed CNN Model Results

The studied models' performances were tested and evaluated using a completely independent data subset already prepared. Before finding the scoring metrics for each performance model, we proceeded with drawing the confusion matrix.  Figure 5 represents the confusion matrix of the five trained models.

From these tables, we noticed that the majority of models give a good classification. However, there is some confusion by some models about the classes of COVID-19 and tuberculosis. However, we can see that the majority of models achieve perfect performance for the four classes. Based on these performances, we moved to the second training level by combining the models' classification. In Figure 6, we represent the confusion matrix of the generated model classification using stacking technique. This matrix gives a performance visualization of the generated model. From this classification, we noticed that the TP is higher compared to the FP and FN for all classes. Moreover, we can observe that the FP and FN of three classes, tuberculosis, viral pneumonia, and normal, are larger compared to the COVID-19 class. This model classified correctly 140 cases as COVID-19, and just 4 cases were classified as COVID-19 although they belong to the tuberculosis class. To understand these experimental results, we employed the confusion matrix results to calculate the evaluation metrics for each model.

To explore these results, we can use a ROC curve to plot the sensitivity versus specificity (or False Positive Rate vs True Positive Rate) of a diagnostic test. Generally, this type of curve helps us to compare several models, according to the value of the AUC variable. This value measures the entire area between two dimensions located under the ROC curve. In this paper, we draw the ROC curve for each model used in this study.  Figure 7 illustrates a plot of the False Positive Rate (FPR) versus True Positive Rate (TPR) for the different classes for the experimented model and proposed model.

From these ROC curves, we can see that all the studied models reached an AUC value of 0.98. It becomes clear that the model based on stacking technique is the best model to classify the X-ray images used in this study. Moreover, we noticed that all the classes achieve a rate of area in the range of 0.99-1. The generated model produced a very high performance compared to the other models. In fact, the proposed model reached an AUC value of 1.00 for COVID-19 class, which has an important clinical advantage.

This means the labeling of COVID-19 cases with other classes is almost zero, which reduces the risk of not detecting COVID-19 cases from their chest X-rays. To clarify these results, Table 10 shows the performance evaluation metrics of the experimented models; the best results are in bold.

From Table 10, we report that most models have a loss value equal to 5.06% except two models: the VGG16 and generated model achieved a loss value equal to 3.69% and 3.09%, respectively. Moreover, the generated model obtained the largest values for all performance metrics computed. This model records the lowest loss value equal to 3.09%. On the other hand, we noticed that the four classifiers ResNet152V2, ResNet101V2, MobileNetV2, and VGG16 reached an accuracy of 98%. However, the VGG19 and the generated model achieved an accuracy of 99.13% and 99.23%, respectively. For the NPV metric, the Base-Models and the proposed model improve a high value of 99.5%.

#### 4.2.3. Runtime Results

The runtime is an important parameter improving the efficiency and the reliability of the system. We compared the required time during the training process of the experimented models. From Table 11, we observe the approximate change in time at the training phase from one model to another. This is mainly due to the total number of parameters for each model. Moreover, when the number of model parameters is high, the time required for the training phase became longer, whether the runtime or the time necessary for each epoch.

### 4.3. Discussion

In this paper, we proposed a novel diagnosis system of COVID-19 based on the stacking technique and TL algorithms. This system aims to find the best diagnostic algorithm for patients infected with COVID-19. The generated model was based on the five TL networks: ResNet152V2, ResNet101V2, MobileNetV2, VGG16, and VGG19. These algorithms were trained and validated on the generated X-ray image dataset from a six-source database. This dataset includes four classes: COVID-19, tuberculosis, viral pneumonia, and normal. At the metamodel level, we used a KNN algorithm to generate a final predictive model. In fact, the KNN algorithm learns how to combine the basic models' predictions and provide the final prediction of patients infected with COVID-19. From the experimental results, we noticed that all the studied models achieve a high accuracy between 98% and 99%. Furthermore, the loss value for most models does not exceed 5%. The graphic presented in Figure 8 summarizes all experimental results presented in this paper.

This graph shows the variation between loss and three scoring metrics: accuracy, precision, and sensitivity. Indeed, when the loss value increases, the values of the three metrics decrease. All models used in this work including the generated model achieved a high value in specificity and NPV metrics. Generally, the proposed diagnostic system showed a high performance compared to other previous works.  Table 12 illustrates a comparison between our proposed system and the other works presented in this paper.

The PCR test is considered by many to be the gold standard for diagnosing COVID-19. Calculating the concordance rate between our method and the PCR test allows us to better judge the potential of our system for prevalent and widespread adoption in the real state of the COVID-19 pandemic. In particular, our system is able to distinguish between four classes: COVID-19, tuberculosis, viral pneumonia, and normal.

## 5. Conclusion and Perspectives

The main contribution of this paper is to propose an efficient pandemic disease diagnostic system. We targeted the COVID-19 diagnostic task from chest X-ray images. The proposed system is based on five basic transfer learning models. Furthermore, the goal was to improve the detection precision of COVID-19 by proposing a new diagnostic tool that combines the performance of TL algorithms to extract the images' features. This allows more stable predictions to be made and improves the learning model. We started by preparing the dataset to be used. We selected the best tested deep learning models from the current state-of-the-art image classification algorithms. We developed their architecture to add our designed head model. We trained all selected classifiers on the processed dataset. We found very encouraging results when testing the test set. All classifiers have an accuracy of about 99%.

To go beyond improving accuracy, we selected the best performing classifiers on the test set. To reinforce our results, we performed the experiments on two different sets (the test set and the validation set). We have found that the best approach to take for COVID-19 diagnosis is the stacking method based on the results given by the studied classifiers: ResNet152V2, ResNet101V2, MobileNetV2, VGG16, and VGG19. The stacking method gave us an average accuracy of 0.9923 with 100% accuracy regarding the COVID-19 class when testing on the test and validation set.

This study places more emphasis on the usefulness of the stacking method in dealing with sensitive and important tasks, such as diagnosing COVID-19.

In future work, we need to invest more in voting approaches by studying their performance on larger datasets. Moreover, we will implement the three ensemble ML methods, using bagging, boosting, and stacking technique. We need to dig deeper into the use of a multilevel stacking technique, to make our system more robust and accurate for diagnosing pandemic or cancerous diseases.

## Figures and Tables

**Figure 1:** Flowchart representing the proposed diagnosis system architecture.

**Figure 2:** Main steps of the stacking technique.

**Figure 3:** X-ray image samples of the 4 classes: (a) COVID-19 sample; (b) tuberculosis sample; (c) viral pneumonia sample; (d) normal sample.

**Figure 4:** Accuracy and loss curves obtained by training and validation Base-Models: (a) ResNet152V2-based model; (b) ResNet101V2-based model; (c) MobileNetV2-based model; (d) VGG16-based model; (e) VGG19-based model.

**Figure 5:** The confusion matrix representing the Base-Models' classification: (a) ResNet152V2-based model; (b) ResNet101V2-based model; (c) MobileNetV2-based model; (d) VGG16-based model; (e) VGG19-based model.

**Figure 6:** The confusion matrix representing the generated model by the stacking technique.

**Figure 7:** ROC curves results for 5 tuned CNN models: (a) ResNet152V2-based model; (b) ResNet101V2-based model; (c) MobileNetV2-based model; (d) VGG19-based model; (e) VGG16-based model. (f) The resulting proposed CNN model obtained by the stacking technique.

**Figure 8:** The performance evaluation metrics for all studied models.

**Table 1:** Summary of related work.

Works	Number of classes	Models used	Accuracy	Precision	Sensitivity	Specificity
[35]	COVID-19	ResNet50	93.01%	95.18%	91.45%	94.77%
	Non-COVID-19					

[36]	COVID-19	CovXNet	90.2%	90.8%	89.9%	89.1%
	Normal					
	Viral pneumonia					
	Bact pneumonia					
	COVID-19		89.6%	88.5%	90.3%	87.6%
	Viral pneumonia					
	Bact pneumonia					

[37]	COVID-19	CoroNet	89.6%	90%	89.92%	96.4%
	Normal					
	Viral pneumonia					
	Bact pneumonia					
	COVID-19		95%	95%	96.9%	97.5%
	Normal					
	Bact pneumonia					

[38]	COVID-19	AlexNet	78.92%	N/A	89.21%	68.63%
		VGG16	83.33%	N/A	80.39%	86.27%
		VGG19	85.29%	N/A	92.16%	78.43%
		SqueezeNet	82.84%	N/A	78.43%	87.52%
		GoogLeNet	85.29%	N/A	81.37%	90.20%
	Viral pneumonia	MobileNetV2	92.16%	N/A	97.06%	87.25%
		ResNet18	91.61	N/A	95.10%	88.23%
		ResNet50	94.12%	N/A	90.20%	100%
		ResNet101	99.51%	N/A	100%	99.02%
		Xception	99.02%	N/A	98.04%	100%

[39]	Normal	VGG16	79.01%	N/A	N/A	N/A
		DenseNet121	89.96%	N/A	N/A	N/A
	COVID-19	Xception	88.03%	N/A	N/A	N/A
		NASNet	85.03%	N/A	N/A	N/A
	Other	EfficientNet	93.48%	N/A	N/A	N/A

[40]	COVID-19	AlexNet	99.13%	N/A	99.47%	99.15%
	Healthy					
	Pneumonia					
	Tuberculosis					

[41]	COVID-19	Majority voting method	99.31%	100%	100%	N/A
	Normal					
	Viral pneumonia					

[42]	COVID-19	DenseNet	97.99%	98.38%	98.15%	N/A
	Normal					
	Pneumonia					

[43]	COVID-19	Majority voting method	99.26%	97.87%	100%	98.89%
	Normal					
	Pneumonia					

[44]	COVID-19	ResNet50V2	95.49%	96.85%	99.19%	98.27%
	Normal	VGG16	92.70%	97.50%	94.35%	98.69%
	Pneumonia	Inception V3	92.97%	97.60%	98.39%	98.67%

[45]	COVID-19	VGG16	91.69%	92.33%	95.92%	100%
	Normal					
	Pneumonia					

[46]	COVID-19	VGG16	87.84%	82.00%	82.33%	91.20%
	Normal	Inception V3	91.32%	87.54%	89.00%	94.00%
	Viral pneumonia	EfficientNetB0	92.93%	88.30%	90.00%	95.00%

**Table 2:** Dataset sources used to generate a combined dataset containing four classes.

Dataset source	COVID-19	Normal	Viral pneumonia	Tuberculosis
COVID-19 Radiography Database (https://www.kaggle.com/tawsifurrahman/covid19-radiography-database/data?select=COVID-19+Radiography+Database)	1200	1341	1345	—
COVID-19 Detection X-Ray Dataset (https://www.kaggle.com/darshan1504/covid19-detection-xray-dataset)	60	880	412	—
COVID-19 Patients Lungs X-Ray Images (https://www.kaggle.com/nabeelsajid917/covid-19-x-ray-10000-images?select=dataset)	70	28	—	—
COVID-19 X-Rays (https://www.kaggle.com/andrewmvd/convid19-x-rays?select=X+rays)	70	—	—	—
Pneumonia Virus vs Pneumonia Bacteria (https://www.kaggle.com/muhammadmasdar/pneumonia-virus-vs-pneumonia-bacteria)	—	—	1493	—
Tuberculosis (TB) Chest X-Ray Database (https://www.kaggle.com/tawsifurrahman/tuberculosis-tb-chest-xray-dataset)	—	—	—	3500
Generated dataset	1400	2249	3250	3500

**Table 3:** Description of the dataset partitions used in this study.

Class	Training (80%)	Validation (10%)	Testing (10%)	Total (100%)
COVID-19	1120	140	140	1400
Tuberculosis	2800	350	350	3500
Viral pneumonia	2600	325	325	3250
Normal	1799	225	225	2249
Total	8319	1040	1040	10399

**Table 4:** The proposed tuned version based on ResNet152V2 model architecture.

Layer type	Output shape	Parameters
resnet152v2 (model)	7 × 7 × 2048	58331648
conv2d_1 (Conv2D)	7 × 7 × 1024	2098176
mp_1 (MaxPooling2D)	3 × 3 × 1024	0
flatten (flatten)	9216	0
dense_1 (dense)	1024	9438208
dense_2 (dense)	512	524800
dense_3 (dense)	256	131328
dense_4 (dense)	4	1028

**Table 5:** The proposed tuned version based on ResNet101V2 model architecture.

Layer type	Output shape	Parameters
resnet101v2 (model)	7 × 7 × 2048	42626560
conv2d_1 (Conv2D)	7 × 7 × 1024	2098176
mp_1(MaxPooling2D)	3 × 3 × 1024	0
flatten (flatten)	9216	0
dense_1 (dense)	1024	9438208
dense_2 (dense)	512	524800
dense_3 (dense)	256	131328
dense_4 (dense)	4	1028

**Table 6:** The proposed tuned MobileNetV2-based model architecture.

Layer type	Output shape	Parameters
mobilenetv2 (model)	7 × 7 × 1280	2257984
conv2d_1 (Conv2D)	7 × 7 × 1024	1311744
mp_1(MaxPooling2D)	3 × 3 × 1024	0
flatten (flatten)	9216	0
dense_1 (dense)	1024	9438208
dense_2 (dense)	512	524800
dense_3 (dense)	256	131328
dense_4 (dense)	4	1028

**Table 7:** The proposed tuned VGG16-based model architecture.

Layer type	Output shape	Parameters
vgg16 (model)	7 × 7 × 512	14714688
conv2d_1 (Conv2D)	7 × 7 × 512	262656
mp_1 (MaxPooling2D)	3 × 3 × 512	0
flatten (flatten)	4608	0
dense_1 (dense)	512	2359808
dense_2 (dense)	256	131328
dense_3 (dense)	4	1028

**Table 8:** Complexity of the proposed tuned VGG19-based model architecture.

Layer type	Output shape	Parameters
vgg19 (model)	7 × 7 × 512	20024384
conv2d_1 (Conv2D)	7 × 7 × 512	262656
mp_1 (MaxPooling2D)	3 × 3 × 512	0
flatten (flatten)	4608	0
dense_1 (dense)	512	2359808
dense_2 (dense)	256	131328
dense_3 (dense)	4	1028

**Table 9:** The best hyperparameters used for the TL models in the training phase.

Network	Learning rate	Batch size	Optimizer	Loss function	Epochs
All Base-Models used in this study	1.000000e-04	16	Adam	Categorical cross entropy	25

**Table 10:** Models' performance evaluation based on scoring metrics: loss, accuracy, precision, sensitivity, specificity, and NPV.

Model	Accuracy (%)	Loss (%)	Precision (%)	Sensitivity (%)	Specificity (%)	NPV (%)
ResNet152V2	98.55	5.06	98.56	98.22	99.5	99.52
ResNet101V2	98.55	5.99	98.32	98.44	99.52	99.51
MobileNetV2	98.36	5.18	98.4	97.99	99.45	99.46
VGG16	98.75	3.69	98.59	98.6	99.59	99.57
VGG19	99.13	5.51	99.27	98.66	99.69	99.73
Generated model by stacking technique	99.23	3.09	98.96	99.34	99.75	99.72

**Table 11:** Description of Base-Models' runtime and time by epoch.

Models	Accuracy (%)	Runtime	Time/epoch (s)	Total parameters (millions)
ResNet152V2	98.55	50 min 33 s	120	70
ResNet101V2	98.55	35 min 21 s	85	54
MobileNetV2	98.36	19 min 50 s	47	13
VGG16	98.75	24 min 27 s	59	17
VGG19	99.13	28 min 55 s	69	22

**Table 12:** Results for the staking technique-based model compared with some previous works.

Works	Methods used	Accuracy	Precision	Sensitivity	Specificity
[35]	ResNet50	93.01%	95.18%	91.45%	94.77%
[36]	CovXNet	89.6%	88.5%	90.3%	87.6%
		90.2%	90.8%	89.9%	89.1%
[37]	CoroNet	95%	95%	96.9%	97.5%
		89.6%	90%	89.92%	96.4%
[38]	AlexNet	78.92%	N/A	89.21%	68.63%
	VGG16	83.33%	N/A	80.39%	86.27%
	VGG19	85.29%	N/A	92.16%	78.43%
	SqueezeNet	82.84%	N/A	78.43%	87.52%
	GoogLeNet	85.29%	N/A	81.37%	90.20%
	MobileNetV2	92.16%	N/A	97.06%	87.25%
	ResNet18	91.61%	N/A	95.10%	88.23%
	ResNet50	94.12%	N/A	90.20%	100%
	ResNet101	99.51%	N/A	100%	99.02%
	Xception	99.02%	N/A	98.04%	100%
[39]	VGG16	79.01%	N/A	N/A	N/A
	DenseNet121	89.96%	N/A	N/A	N/A
	Xception	88.03%	N/A	N/A	N/A
	NASNet	85.03%	N/A	N/A	N/A
	EfficientNet	93.48%	N/A	N/A	N/A
[40]	AlexNet	99.13%	N/A	99.47%	99.15%
[41]	Majority voting method	99.31%	100%	100%	N/A
[42]	DenseNet	97.99%	98.38%	98.15%	N/A
[43]	Majority voting method	99.26%	97.87%	100%	98.89%
[44]	ResNet50V2	95.49%	96.85%	99.19%	98.27%
	VGG16	92.70%	97.50%	94.35%	98.69%
	Inception V3	92.97%	97.60%	98.39%	98.67%
[45]	VGG16	91.69%	92.33%	95.92%	100%
[46]	VGG16	87.84%	82.00%	82.33%	91.20%
	Inception V3	91.32%	87.54%	89.00%	94.00%
	EfficientNetB0	92.93%	88.30%	90.00%	95.00%
**Proposed model**	**Stacking technique**	**99.23% [95% CI: 98.3–100]**	**98.96% [95% CI: 98–100]**	**99.34% [95% CI: 98.4–100]**	**99.75% [95% CI: 98.5–100]**

The bold values mean the performance evaluation metrics obtained with our proposed model based on stacking technique. The values between lead to the confidence interval (CI) that is the standard used to quantify the uncertainty of estimating the obtained performance evaluation metrics.

## Data Availability

The data used to support the results are available from the corresponding author upon reasonable request.
